RETRACTED

# miR-139-5p Inhibits Lung Adenocarcinoma Cell Proliferation, Migration, and Invasion by Targeting MAD2L1

**DOI:** 10.1155/2020/2953598

**Published:** 2020-11-04

**Authors:** Jianfeng Li, Xi He, Xiaotang Wu, Xiaohui Liu, Yixiong Huang, Yuchen Gong

**Affiliations:** ^1^Department of Thoracic Surgery, Tangshan People's Hospital, Tangshan, China; ^2^Shanghai Engineering Research Center of Pharmaceutical Translation, Shanghai, China; ^3^Department of Thoracic Surgical Oncology, Fujian Cancer Hospital & Fujian Medical University Cancer Hospital, Fujian, China; ^4^Department of Respiration, China Coast Guard of the Chinese People's Armed Police Force Hospital, Zhejiang Province, China

## Abstract

**Background:**

miR-139-5p is lowly expressed in various human cancers and exerts its antitumor effect through different molecular mechanisms, yet the molecular mechanism of miR-139-5p in lung adenocarcinoma (LUAD) remains to be further elucidated. The study is aimed at investigating the role and the regulatory mechanism of miR-139-5p in LUAD progression.

**Methods:**

Differential analysis was performed on miRNA expression data in the TCGA-LUAD dataset. qRT-PCR was employed to detect the transcription levels of miR-139-5p and MAD2L1 in LUAD cells, while western blot was carried out for the detection of MAD2L1 protein expression. CCK-8 and Transwell assays were implemented to assess LUAD cell proliferation, migration, and invasion. A dual-luciferase reporter gene assay was conducted to verify the direct targeting relationship between miR-139-5p and MAD2L1.

**Results:**

miR-139-5p was significantly downregulated in LUAD cells in comparison with that in human normal bronchial epithelial cells. Overexpressing miR-139-5p inhibited LUAD cell proliferation, migration, and invasion, while opposite results could be observed when miR-139-5p was inhibited. MAD2L1 was identified as a direct target of miR-139-5p in LUAD. Besides, the inhibitory effect of miR-139-5p overexpression on LUAD cell proliferation, migration, and invasion was attenuated by overexpressing MAD2L1.

**Conclusion:**

Our study suggests that miR-139-5p is lowly expressed in LUAD cells and inhibits LUAD cell proliferation, migration, and invasion by targeted suppressing MAD2L1 expression. It is of potential significance for the prognosis and treatment of LUAD.

## 1. Introduction

Lung adenocarcinoma (LUAD), the most common type of nonsmall cell lung cancer (NSCLC), is characterized by dense lymphocyte infiltration and is prone to metastasize at early stages [1]. Different medical interventions, such as chemotherapy, surgical removal, and radiotherapy, are the conventional treatments for LUAD. However, these treatments lack specificity and will also do harm to adjacent normal cells [2], which make the treatment for LUAD evolve from cytotoxic chemotherapy to personalized treatment based on molecular alterations [3]. In recent years, the identification of oncogenes and the use of immunotherapy have already changed the treatment strategies for LUAD, but the survival rate still remains low [4]. Therefore, it is of paramount importance to find a novel therapeutic target to improve the treatment for LUAD.

RETRACTED

Noncoding RNAs have always been a hot topic in the cancer field for years, especially microRNAs (miRNAs). The reason is that they are key players in mediating different molecular processes and they participate in tumorigenesis more often than protein-coding genes [5]. miRNAs are involved in the control of several cancer-related processes, such as proliferation, apoptosis, migration, and invasion. Additionally, miRNAs are also involved in many other diseases, such as metabolic disorders [6]. miR-197-3p, as reported, serves as an oncogene in LUAD to promote LUAD cell proliferation and inhibit cell apoptosis by downregulating lysine 63 deubiquitinase (CYLD) [7]. miR-938 exerts its cancer-promoting role in LUAD by targeting RBM5 [8]. As a tumor suppressor, miR-144-3p inhibits LUAD cell proliferation and invasion by increasing the EZH2 expression [9]. These findings indicate that miRNAs have a great potential in the diagnosis and targeted therapy of LUAD.

It is reported that miR-139-5p is downregulated in various cancers and exerts its antitumor role by different molecular mechanisms. For example, miR-139-5p plays an antitumor role in cervical cancer and inhibits Wnt/*β*-catenin signal transduction by targeting transcription factor 4 (TCF4) [10]. In oral squamous cell carcinoma, miR-139-5p inhibits cell proliferation and metastasis by suppressing HOXA9 expression [11]. Moreover, miR-139-5p acts as a tumor suppressor by regulating SOX5 in prostate cancer cells [12]. However, the mechanism of miR-139-5p underlying LUAD cell proliferation, migration, and invasion remains to be improved and supplemented.

In this study, we made an attempt to explore the expression and role of miR-139-5p in LUAD and the underlying molecular mechanism of miR-139-5p in regulating LUAD cell proliferation, migration, and invasion. Our study may bring additional insights into the molecular mechanism underlying LUAD progression and provide potential indicators for the diagnosis and prognosis of LUAD.

## 2. Materials and Methods

### 2.1. Bioinformatics Analysis

Expression data of miRNAs and mRNAs of the TCGA-LUAD dataset were downloaded from the TCGA database (https://portal.gdc.cancer.gov/), of which miRNA expression data were obtained from 46 normal tissue samples and 521 tumor tissue samples, and mRNA expression data were obtained from 59 normal tissue samples and 535 tumor tissue samples. Expression analysis was performed on miR-139-5p according to the obtained data. Differential analysis was carried out using “edgeR” package with threshold set as ∣logFC | >2.0, *p* < 0.01, and then differentially expressed mRNAs (DEmRNAs) were obtained. Three databases miRDB (http://mirdb.org/), miDIP (http://ophid.utoronto.ca/mirDIP/index.jsp#r), and starBase (http://starbase.sysu.edu.cn/) were employed to predict the target genes of miR-139-5p. Candidate genes obtained from the intersection of DEmRNAs and predicted target genes of miR-139-5p were subjected to Pearson correlation analysis, and the mRNA showing the highest negative correlation coefficient was selected as the object of the study.

RETRACTED

### 2.2. Cell Culture

LUAD cell lines A549 (BNCC337696), PC-9 (BNCC340767), H1975 (BNCC340345), H1650 (BNCC100260), and human normal bronchial epithelial cell line BEAS-2B (BNCC338205) were all purchased from BeNa Culture Collection (Beijing, China). All cell lines were cultured in 100 U RPMI-1640 mediums supplemented with 10% fetal bovine serum (FBS), 100 U/ml penicillin (Invitrogen, Grand Island, NY, USA), and 100 *μ*g/ml streptomycin (Invitrogen, Grand Island, NY, USA), and maintained in an incubator with 5% CO_2_ at 37°C.

### 2.3. Cell Transfection

miR-139-5p mimic, miR-139-5p inhibitor, oe-MAD2L1, and their corresponding negative controls (NC) were accessed from RiboBio (Guangzhou, China). Cells were grown in antibiotic-free complete mediums 24 h before transfection. Lipofectamine 2000 (Thermo Fisher Scientific, Inc.) was employed to transfect cells at a concentration of 50 nM according to the manufacturer's protocol.

### 2.4. qRT-PCR

After 48 h of transfection, total RNA was extracted from LUAD cells using a Trizol kit (Invitrogen Life Technologies, Carlsbad, CA, USA). miRNA and mRNA were reversely transcribed into cDNA by the PrimeScript RT kit (Takara, Japan). qRT-PCR was performed by SYBR Premix Ex Taq (Takara) under the Applied Biosystems ABI 7500 Real-Time PCR System (Thermo Fisher Scientific, Inc.). Primers were shown in Table 1. U6 and GAPDH were applied as endogenous references of miRNA and mRNA, respectively. The relative expression was analyzed by the 2^-*ΔΔ*Ct^ method.

### 2.5. Western Blot

Transfected cells were washed with phosphate-buffered saline (PBS) twice and then were lysed on ice with RIPA loading buffer (Thermo Fisher Scientific, MA, USA) containing protease and phosphatase inhibitor (Solarbio). Protein concentration was assayed by the BCA kit (Beyotime). The protein samples were separated by 10% sodium dodecyl sulfate-polyacrylamide gel electrophoresis (SDS-PAGE; 50 *μ*g/lane) and then transferred onto polyvinylidene fluoride (PVDF) membranes (ZY-160FP, Zeye Bio Co., Ltd., Shanghai, China). After being blocked with 5% skim milk for 2 h at 37°C and washed with Tris-Buffered Saline Tween (TBST) three times, the membranes were incubated with rabbit polyclonal anti-MAD2L1 antibody (1 : 1000, ab97777, Abcam, Cambridge, UK) at 4°C overnight. Rabbit monoclonal anti-GAPDH antibody (1 : 2500, ab9485, Abcam, Cambridge, UK) was taken as control. After being washed with TBST, the membranes were incubated with goat anti-rabbit IgG H&L (1 : 2000, ab205718, Abcam, Cambridge, UK) for 2 h. Finally, protein bands were visualized using an electrochemiluminescence kit (ECL; Pierce Biotechnology) and analyzed by imaging system (ZG11SCIBRIGHTCL, Bio-Rad, CA, USA).

RETRACTED

### 2.6. CCK-8

Cell-counting kit-8 (CCK-8) assay was used for detection of cell proliferation in different transfection groups. Cells (2 × 10^3^) were seeded into 96-well plates (Corning Costar, Corning, NY), and then 10 *μ*l of CCK-8 solution (Beyotime, Nanjing, Jiangsu, China) was added into plates at 0 h, 24 h, 48 h, and 72 h for 2 h of incubation, respectively. The absorbance at 450 nm was measured by an enzyme-labeled instrument (BioTek Company, Winooski, VT, USA) to evaluate cell viability.

### 2.7. Colony Formation Assay

After 24 h of transfection, A549 cells were inoculated into a 6-well plate with 1 × 10^3^ cells/well, and each treatment group was made in triplicate. Cells were cultured in a complete medium for one week until clear colonies were formed. Cell colonies were fixed with 70% methanol for 5 min and stained with 0.5% crystal violet (Thermo Fisher, USA). Each well was washed with sterile water to remove residual crystal violet. Colonies with more than 50 cells were identified, and the number of colonies per well was calculated.

### 2.8. Transwell Migration and Invasion Assays

Transwell assay was applied to evaluate cell migration and invasion. Trypsinized cells were collected after 48 h of transfection. For cell invasion assay, 88 *μ*m pore size inserts (Transwell; Costar, High Wycombe, UK) were placed into 24-well plates to separate the upper chambers from the lower chambers. A total of 200 *μ*l cell suspension containing (3–5) ×10^4^ cells was added into the upper chambers precoated with Matrigel (BD Biosciences, San Jose, CA, USA). 500 *μ*l RPMI-1640 medium supplemented with 20% FBS was added into the lower chambers. Cells invading the lower chambers were then fixed with 70% methanol and treated by 0.5% crystal violet after 24 h. The invaded cells were counted under an inverted microscope (Olympus IX83; Olympus Corporation, Tokyo, Japan). The procedure of cell migration assay was similar to the invasion assay, except that the upper chambers were not precoated with Matrigel.

RETRACTED

### 2.9. Dual-Luciferase Reporter Gene Assay

Amplified wild type (WT) and mutant (MUT) MAD2L1 3′UTR were accessed from Shanghai GenePharma Co., Ltd. and inserted into luciferase vector PmirGLO. PmirGLO-MAD2L1-Wt/PmirGLO-MAD2L1-Mut and miR-139-5p mimic/NC mimic were cotransfected into LUAD cell lines by using Lipofectamine™2000 kit (Invitrogen). After 48 h of transfection, the relative activity of luciferase was assayed by dual-luciferase reporter gene system (Promega Corporation) according to the manufacturer's instructions.

### 2.10. Statistical Analysis

All data were analyzed by GraphPad Prism 6.0 (La Jolla, CA). Each experiment was repeated three times. The results were presented by means ± standard deviation (SD). Student's *t*-test was used for comparison between two groups. *p* < 0.05 was considered statistically significant.

## 3. Results

### 3.1. miR-139-5p Is Downregulated in LUAD Cells

miR-139-5p expression was searched in the TCGA-LUAD dataset, and it was found that miR-139-5p was significantly downregulated in LUAD tissues (Figure 1(a)). qRT-PCR was employed to detect the expression of miR-139-5p in LUAD cell lines A549, PC-9, H1975, H1650, and human normal bronchial epithelial cell line BEAS-2B, exhibiting that the expression of miR-139-5p was remarkably downregulated in LUAD cell lines relative to that in human normal bronchial epithelial cell line (Figure 1(b)). A549 cell line with the lowest expression level of miR-139-5p was selected for subsequent experiments.

### 3.2. miR-139-5p Inhibits LUAD Cell Proliferation, Migration, and Invasion

To verify the biological function of miR-139-5p in LUAD, miR-139-5p mimic or miR-139-5p inhibitor and their corresponding NC were transfected into A549 cells for evaluation of cell proliferation, migration, and invasion. First of all, qRT-PCR was used to detect the expression level of miR-139-5p in different groups, and the results displayed that the expression of miR-139-5p after transfection met the requirements (Figure 2(a)), and the successfully transfected cells could be used in subsequent experiments. Cell biological behaviors in each group were sequentially assayed. As revealed by CCK-8, we found that the viability of A549 cells transfected with miR-139-5p mimic was markedly lower than that of A549 cells transfected with NC mimic, while the cell proliferative ability was significantly increased in the miR-139-5p inhibitor than that in the NC inhibitor group (Figure 2(b)). The results of colony formation assay indicated that the colony formation ability of miR-139-5p overexpressed cells was significantly inhibited, while that of LUAD cells was remarkably improved after miR-139-5p was inhibited (Figure 2(c)). Next, the Transwell assay illustrated that the migration and invasion of A549 cells transfected with miR-139-5p mimic were considerably inhibited, while those of A549 cells transfected with miR-139-5p inhibitor were increased (Figures 2(d) and 2(e)). Collectively, these findings suggested that miR-139-5p inhibited A549 cell proliferation, migration, and invasion as a tumor suppressor in LUAD.

RETRACTED

### 3.3. MAD2L1 Is a Direct Target of miR-139-5p

We then explored the underlying molecular mechanism of miR-139-5p in LUAD. Databases including miRDB, miDIP, and starBase were firstly implemented for target prediction for miR-139-5p, and five candidate genes (NPTX1, ELAVL2, FBN2, GPR37, and MAD2L1) obtained from the intersection of predicted genes and upregulated DEmRNAs were subjected to Pearson correlation analysis with miR-139-5p. The result showed that MAD2L1 had the highest negative correlation coefficient with miR-139-5p (Figures 3(a)–3(c)). Expression analysis was performed on MAD2L1 in the TCGA-LUAD dataset, which discovered that MAD2L1 was noticeably highly expressed in LUAD tissue, and LUAD patients with high MAD2L1 expression had relatively low overall survival (OS) (Figures 3(d) and 3(e)). We speculated that MAD2L1 might be a direct target of miR-139-5p based on the result of bioinformatics analysis.

To validate our speculation, miR-139-5p mimic or miR-139-5p inhibitor and their corresponding NC were firstly transfected into A549 cells, and then qRT-PCR and western blot were conducted to determine the transcription level and protein expression level of MAD2L1. The results indicated that the mRNA and protein expression levels of MAD2L1 were significantly downregulated after miR-139-5p was overexpressed, whereas opposite results were observed when miR-139-5p was suppressed (Figures 3(f) and 3(g)). Furthermore, the binding sites of miR-139-5p on MAD2L1 3′UTR were predicted by the starBase database (Figure 3(h)) and then verified by dual-luciferase assay. We found that the luciferase activity of A549 cells transfected with miR-139-5p mimic and MAD2L1-Wt was decreased, while that of A549 cells cotransfected with miR-139-5p mimic and MAD2L1-Mut exhibited no marked change (Figure 3(i)). Taken together, these findings elucidated that MAD2L1 was a direct target of miR-139-5p and was negatively regulated by miR-139-5p.

### 3.4. MAD2L1 Mediates the Effect of miR-139-5p on LUAD Cells

To investigate whether miR-139-5p inhibited LUAD cell proliferation, migration, and invasion by regulating MAD2L1, we designed three groups: NC mimic+oe-NC, miR-139-5p mimic+oe-NC, and miR-139-5p mimic+oe-MAD2L1. We found that the inhibitory effect of miR-139-5p overexpression on MAD2L1 expression could be reversed by overexpressing MAD2L1 (Figures 4(a) and 4(b)). CCK-8 and colony formation assays suggested that the overexpression of miR-139-5p significantly inhibited the proliferation of LUAD cells, while the overexpression of MAD2L1 reversed the inhibitory effect of miR-139-5p on cell proliferation (Figures 4(c) and 4(d)). Transwell assay was conducted for testing cell migration and invasion. The results illustrated that overexpressing miR-139-5p markedly inhibited cell migration and invasion, whereas overexpressing MAD2L1 reversed the inhibitory effect of miR-139-5p on cell behaviors (Figures 4(e) and 4(f)). Therefore, miR-139-5p inhibited LUAD cell proliferation, migration, and invasion by regulating MAD2L1.

RETRACTED

## 4. Discussion

miRNAs are capable of interfering transcriptional signal transduction and regulating the key processes of cells, thus playing vital roles in the occurrence and development of cancers [13]. It has been reported that the differential expression of miRNAs between normal lung and cancerous lung leads to the emergence of novel biomarkers, which is conducive to the screening of high-risk groups and helps the diagnosis and treatment of lung cancer [14]. Up to now, the potential miRNAs that regulate the progression of LUAD have not been fully identified.

In this study, miR-139-5p expression was searched in the TCGA-LUAD dataset, finding that miR-139-5p was downregulated in LUAD tissue. miR-139-5p was lowly expressed in LUAD cell lines as evidenced by qRT-PCR, and the result was consistent with the expression of miR-139-5p in hepatocellular carcinoma (HCC) [15], endometrial carcinoma [16], and gallbladder carcinoma [17]. In osteosarcoma, overexpressing miR-139-5p inhibits cell proliferation, migration, and invasion, while loss of miR-139-5p facilitates cell proliferation, migration, and invasion [18], and similar trends could be observed in LUAD in this study. These findings indicate that miR-139-5p acts as a tumor suppressor in LUAD.

Due to the fact that miRNAs can regulate the growth and metastasis of tumor by various molecular mechanisms [19], we performed bioinformatics analysis to predict the target gene of miR-139-5p, and MAD2L1 was identified as a potential target of miR-139-5p. A dual-luciferase reporter gene assay was conducted and confirmed the targeting relationship between the two genes. Besides, MAD2L1 was found to be highly expressed in LUAD tissue, and LUAD patients with high MAD2L1 expression had relatively low OS, which were consistent with the results of the study made by Li et al. regarding to MAD2L1 expression in HCC [20]. MAD2L1 is reported to be a key player in maintaining the function of spindle assemble checkpoint. The overexpression of MAD2L1 in spindle assemble checkpoint can result in the instability and aneuploidy of chromosome, and the genetic variation of MAD2L1 can lead to lung cancer susceptibility [21, 22]. Therefore, we further confirmed whether miR-139-5p exerted its antitumor role in LUAD by suppressing MAD2L1. miR-139-5p and MAD2L1 were simultaneously overexpressed in LUAD cells, and we found that the inhibitory effect of miR-139-5p overexpression on cell proliferation, migration, and invasion was reversed by MAD2L1 overexpression. Hence, we believed that miR-139-5p regulated LUAD cell proliferation, migration, and invasion by targeting MAD2L1.

RETRACTED

Generally speaking, we elucidated that miR-139-5p was lowly expressed in LUAD and inhibited LUAD cell proliferation, migration, and invasion. Besides, MAD2L1 was identified as a direct target of miR-139-5p in LUAD, and miR-139-5p exerted its antitumor role by inhibiting MAD2L1 expression. Our discovery not only lays a molecular foundation for exploration of the mechanism of miR-139-5p in LUAD but also provides a potential target for the treatment of LUAD.

## Figures and Tables

**Figure 1:** miR-139-5p is downregulated in LUAD cells. (a) Box plots of miR-139-5p expression in the TCGA-LUAD dataset; (b) The expression level of miR-139-5p in LUAD cell lines A549, PC-9, H1975, H1650, and human normal bronchial epithelial cell line BEAS-2B was detected by qRT-PCR; ^∗^*p* < 0.05.

**Figure 2:** miR-139-5p inhibits LUAD cell proliferation, migration, and invasion. (a) qRT-PCR was used to detect the transfection efficiency of miR-139-5p in A549 cells; (b) CCK-8 was performed for the detection of cell viability in different transfection groups; (c) Colony formation assay was performed to detect the colony formation ability of A549 cells in different transfection groups; (d, e) Transwell assay (100×) was carried out for assessment of cell (d) migration and (e) invasion in each transfection group; ^∗^*p* < 0.05.

**Figure 3:** miR-139-5p targeted binds to MAD2L1 and negatively regulates MAD2L1 expression. (a) Venn diagram of target genes of miR-139-5p predicted by miRDB, miDIP, and starBase databases and upregulated DEmRNAs in the TCGA-LUAD; (b) Pearson correlation of miR-139-5p and five candidate genes NPTX1, ELAVL2, FBN2, GPR37, and MAD2L1; (c) Pearson correlation of miR-139-5p and MAD2L1; (d) Box plots of MAD2L1 expression in LUAD tissue and normal tissue in the TCGA-LUAD dataset; (e) Survival curves of patients with high expression of MAD2L1 (red) and low expression of MAD2L1 (blue). The abscissa refers to the time (in years) and the ordinate refers to survival rate; (f) qRT-PCR was used to detect the mRNA expression level of MAD2L1 after transfection of miR-139-5p mimic or miR-139-5p inhibitor; (g) Western blot was employed to examine the protein expression of MAD2L1 after transfection; (h) starBase database was used to predict the binding sites of miR-139-5p on MAD2L1 3′UTR; (i) Dual-luciferase reporter gene assay was used for verification of the targeted binding relationship between miR-139-5p and MAD2L1; ^∗^*p* < 0.05.

RETRACTED

**Figure 4:** MAD2L1 mediates the effect of miR-139-5p on LUAD cells. (a, b) qRT-PCR and western blot were carried out to assess the mRNA and protein expression of MAD2L1 in each treatment group; (c, d) CCK-8 and colony formation assays were conducted for the assessment of cell proliferation in different treatment groups; (e, f) Transwell assay (100×) was performed to assess (e) cell migration and (f) invasion in different treatment groups; ^∗^*p* < 0.05.

**Table 1:** Primer sequences in qRT-PCR.

Gene	Forward	Reverse
miR-139-5p	5′-TCTACAGTGCACGTGTCTCCA G-3′	5′-GTGCAGGGTCCGAGGT-3′
U6	5′-TGCGGG TGCTCGCTTCGGCAG C-3′	5′-GTGCAGGGTCCGAGGT-3′
MAD2L1	5′-GTTCTTCTCATTCGGCATCAACA-3′	5′-GAGTCCGTATTTCTGCACTCG-3′
GAPDH	5′-GGAGCGAGATCCCTCCAAAAT-3′	5′-GGCTGTTGTCATACTTCTCATGG-3′

## Data Availability

The data and materials in the current study are available from the corresponding author on reasonable request.
